The article "Enpp1: A Potential Facilitator of Breast Cancer Bone Metastasis" was published in 2013. Journal: PLoS One.

# Enpp1: A Potential Facilitator of Breast Cancer Bone Metastasis

**DOI:** 10.1371/journal.pone.0066752

**Published:** 2013-07-05

**Authors:** Wen Min Lau, Michele Doucet, Ryan Stadel, David Huang, Kristy L. Weber, Scott L. Kominsky

**Affiliations:** Department of Orthopaedic Surgery, Johns Hopkins University School of Medicine, Baltimore, Maryland, United States of America; Sanford Burnham Medical Research Institute, United States of America

## Abstract

Bone is the most common site of breast cancer metastasis and once established, it is frequently incurable. Critical to our ability to prevent and treat bone metastasis is the identification of the key factors mediating its establishment and understanding their biological function. To address this issue we previously carried out an *in vivo* selection process to isolate murine mammary tumor sublines possessing an enhanced ability to colonize the bone. A comparison of gene expression between parental cells and sublines by genome-wide cDNA microarray analysis revealed several potential mediators of bone metastasis, including the pyrophosphate-generating ectoenzyme Enpp1. By qRT-PCR and Western analysis we found that expression of Enpp1 was elevated in human breast cancer cell lines known to produce bone metastasis in animal models compared to non-metastatic and normal mammary epithelial cell lines. Further, in clinical specimens, levels of Enpp1 were significantly elevated in human primary breast tumors relative to normal mammary epithelium, with highest levels observed in breast-bone metastasis as determined by qRT-PCR and immunohistochemical analysis. To examine the potential role of Enpp1 in the development of bone metastasis, Enpp1 expression was stably increased in the breast cancer cell line MDA-MB-231 and the ability to colonize the bone following intracardiac and direct intratibial injection of athymic nude mice was determined. By both routes of administration, increased expression of Enpp1 enhanced the ability of MDA-MB-231 cells to form tumors in the bone relative to cells expressing vector alone, as determined by digital radiography and histological analysis. Taken together, these data suggest a potential role for Enpp1 in the development of breast cancer bone metastasis.

## Introduction

Metastasis is the ultimate cause of mortality in breast cancer patients, developing in the bone more frequently than any other site. Bone metastasis occurs in approximately 80% of patients with advanced breast cancer and causes considerable morbidity in the form of bone pain, pathological fractures, nerve compression, and life-threatening hypercalcemia. Sadly, bone metastasis is frequently incurable and the median survival time following diagnosis is just 2 years. Despite ongoing research efforts, the molecular and cellular mechanisms that regulate the development of bone metastasis and resultant osteolysis remain poorly understood. Identification of factors regulating this process may reveal novel targets for preventative and therapeutic interventions against this devastating disease.

In this study, we identified the ectoenzyme ectonucleotide pyrophosphatase/phosphodiesterase I (Enpp1) as being overexpressed in human primary breast cancer relative to normal mammary epithelium and provide the first evidence of its potential to foster the development of bone metastasis. Enpp1 is a type II transmembrane glycoprotein with pyrophosphatase and phosphodiesterase activity, expressed highly in bone and cartilage [1]. *Enpp1* is located at 6q22-q23, a region reportedly amplified in breast cancer [2], [3], and its mutation has been associated with several disorders including infantile arterial calcification [4], [5], ossification of the posterior longitudinal ligament of the spine [6], and insulin resistance [7]. Biologically, Enpp1 is well known for its role in regulating bone mineralization, serving as the principal ectoenzyme responsible for the generation of extracellular inorganic pyrophosphate (PP_i_) [1], a potent inhibitor of hydroxyapatite formation [8], [9]. In addition, Enpp1 has been shown to modulate insulin signaling, recently reported to regulate bone acquisition and energy metabolism through effects on osteoblasts [10], while also functioning in purinergic signaling [11].

## Results and Discussion

### Association of Enpp1 with Breast Cancer Bone Metastasis

Previously, we utilized the murine mammary tumor cell line NT2.5 in an *in vivo* selection process to generate sublines having an increased propensity to develop metastasis to bone as compared to other sites [12]. To identify genes potentially important for the development of bone metastasis, microarray analysis was conducted comparing gene expression between parental NT2.5 cells and sublines having a moderately (BO3) and highly (BO6) increased preference for the colonization of bone following intracardiac injection. These microarray data have been deposited in the National Center for Biotechnology Information (NCBI) Gene Expression Omnibus (GEO) under accession number GSE47714. While many candidates were identified in this analysis [12], of particular interest was the pyrophosphate-generating ectoenzyme Enpp1, a central regulator of extracellular PP_i_ levels, which have a substantial impact on bone physiology [13]. By microarray analysis, Enpp1 mRNA levels were incrementally increased from parental NT2.5 cells to BO3 and finally BO6 sublines (*p* = 0.008), which was confirmed in a separate experiment by qRT-PCR (Fig. 1A).

**Figure 1:** Expression of Enpp1 in breast cancer cell lines. Enpp1 (**A, B**) mRNA and (**C**) protein expression was determined in (A) NT2.5 murine breast cancer cells and bone sublines, and (B, C) immortalized normal human mammary epithelial cell lines and human breast cancer cell lines by (A, B) qRT-PCR and (C) Western analysis. (A, B) Data are representative of three independent experiments performed in triplicate and expressed as the mean ± s.e.m (**p<0.01, ***p<0.001). (C) Protein expression was determined by Western analysis performed on equal amounts of protein from total cell lysates.

### Expression of Enpp1 in Human Breast Cancer Cell Lines and Tissues

To determine whether the expression pattern of Enpp1 observed using the NT2.5 murine mammary tumor model translated to human breast cancer, we examined the expression of Enpp1 in a panel of human breast cancer cell lines with and without the ability to establish bone metastasis in animal models (our unpublished observations). Similar to our observation in NT2.5 cells and bone metastasis sublines, Enpp1 expression was elevated in human breast cancer cell lines that are capable of forming bone metastasis in animal models (MDA-MB-231/MDA-MB-468) as compared to those incapable of colonizing the bone (MCF-7/SKBR3), which displayed expression levels similar to that in immortalized normal mammary epithelial cell lines (MCF-10A/HBL-100) (Fig. 1B, C). Extending our investigation to clinical samples, we found that Enpp1 mRNA expression was significantly elevated in primary breast tumors relative to normal mammary epithelium (*p*<0.05), with the highest levels observed in breast-bone metastasis (Fig. 2A). Correspondingly, immunohistochemical (IHC) analysis revealed strong Enpp1 protein expression in 32% (n = 37) of primary breast tumors while little to no Enpp1 expression was detected in adjacent normal mammary epithelium (Fig. 2B, C). Further, Enpp1 was strongly expressed in 100% (n = 6) of breast-bone metastases (Fig. 2D). Importantly, the results of our IHC analysis not only correlated with our mRNA findings, but confirmed that Enpp1 was expressed in tumor cells as opposed to other cell types within these tissues.

**Figure 2:** Expression of Enpp1 in human primary breast cancer and bone metastasis tissues. Enpp1 (**A**) mRNA and (**B–D**) protein expression in human normal mammary epithelium (N), primary breast tumor (T), and breast cancer bone metastasis (BBM) was determined by (A) qRT-PCR and (B–D) IHC analysis. (A) Data are representative of three independent experiments performed in triplicate (*p<0.05 for T versus N). (B–D) Proteins were identified using DAB (brown). Sections were counterstained with hematoxylin and visualized by light microscopy (200X). N – Normal, T – Tumor.

### Effect of Enpp1 on the Establishment of Bone Metastasis

To investigate the potential importance of Enpp1 in the establishment of bone metastasis, we utilized the MDA-MB-231 breast cancer cell line, which is capable of forming osteolytic bone metastasis in animal models and displayed moderate expression of Enpp1 by Western analysis (Fig. 1C). MDA-MB-231 cells were stably infected with a retroviral expression vector containing full-length Enpp1 cDNA or with vector alone (EV). Levels of biologically active Enpp1 were increased by greater than two-fold as determined by Western analysis (Fig. 3A) and nucleotide phosphodiesterase activity assay (Fig. 3B). Further, the rate of cell proliferation in MDA-MB-231-Enpp1 cells was equivalent to that in MDA-MB-231-EV cells as determined by MTS assay (data not shown). It should be noted that in an attempt to compliment this gain-of-function approach with a loss-of-function approach employing RNAi, we observed that all control shRNA tested, whether scrambled Enpp1 sequence or unrelated sequence, resulted in reduced Enpp1 expression, preventing use of this strategy and indicating that Enpp1 may be subject to off-target RNAi effects.

**Figure 3:** Generation of breast cancer cells with increased Enpp1 expression and enzymatic activity. MDA-MB-231 cells were stably transduced with Enpp1 or empty vector (EV). Enpp1 (**A**) protein expression was determined by Western analysis performed on equal amounts of protein from total cell lysates. (**B**) Nucleotide phosphodiesterase activity was determined using the nucleotide derivative p-nitrophenyl thymidine 5′-monophosphate (pNP-TMP) as a substrate. Data are representative of three independent experiments performed in triplicate and expressed as the mean ± s.e.m (**p<0.01).

To determine whether increased levels of Enpp1 influence the formation of bone metastasis *in vivo*, both intratibial and intracardiac xenograft model systems were used. As expected, both the MDA-MB-231-Enpp1 and MDA-MB-231-EV group displayed a 100% overall incidence of bone metastasis. However, following both intratibial and intracardiac tumor cell administration, animals that received MDA-MB-231-Enpp1 cells demonstrated more rapid disease progression, evidenced by a significant increase in both osteolysis and tumor area as measured on radiographic images (Fig. 4A, C) and histological sections (Fig. 4 B, D), respectively. Taken together, these data indicate that increased expression of Enpp1 can enhance the development of bone metastasis.

**Figure 4:** Effect of Enpp1 on the development of bone metastasis. MDA-MB-231 cells stably expressing Enpp1 or empty vector (EV) were injected into the (**A, B**) tibia (n = 9/group) and (**C, D**) left cardiac ventricle (n = 5/group) of athymic nude mice and digital radiographic imaging was performed at weekly intervals. (A, C) Osteolytic area and (B, D) tumor area were measured on radiographic images and histological sections, respectively (*p<0.05, **p<0.01). Representative images are shown at 4 weeks following tumor cell administration. Black outlined areas on histological images indicate areas of tumor.

Although the mechanism through which Enpp1 enhances the development of osteolytic bone metastasis remains unknown, given its function as a nucleotide pyrophosphatase/phosphodiesterase, it may be linked to the production of extracellular inorganic pyrophosphate. The balance of PP_i_ and inorganic phosphate (P_i_) is critical to bone physiology, as PP_i_ acts as an inhibitor of mineral deposition [14], [15]. In addition, PP_i_ has been shown to increase production of osteopontin in osteoblasts, another key mineralization inhibitor [16]. In the case of bone metastasis, it is possible that levels of PP_i_ within the bone environment become elevated by the presence of tumor cells expressing Enpp1. This imbalance in PP_i_ could lead to reduced mineralization, potentially creating an environment favoring bone resorption, which has been shown to be critical to the development of bone metastasis as it liberates growth factors from the bone, fueling tumor growth [17]. Beyond its effects on PP_i_/P_i_ balance, the involvement of Enpp1 in insulin and purinergic signaling represent additional avenues worthy of investigation, all having the potential to yield novel insights regarding the interaction between tumor cells and the bone environment.

In summary, we have provided evidence that Enpp1 expression is elevated in human primary breast tumors relative to normal mammary epithelium, with highest levels observed in breast-bone metastasis. Further, consistent with the expression patterns observed in both murine and human breast cancer cell lines, increased expression of Enpp1 enhanced the development of bone metastasis in animal models. These data not only support a potential role for Enpp1 in breast-bone metastasis, but suggest that Enpp1 may be useful as a prognostic indicator for breast cancer.

## Materials and Methods

### Ethics Statement

All experiments were carried out in accordance with the National Research Council's “Guide to the Care and Use of Laboratory Animals”. Animal use was approved by the Johns Hopkins Animal Care and Use Committee, animal welfare assurance #A3272-01, protocol #MO10M450.

### Cell lines and tissues

The murine mammary carcinoma cell line NT2.5 and sublines, BO3 and BO6, were obtained as previously described [12]. NT2.5 parental cells and sublines were maintained in RPMI supplemented with 20% fetal bovine serum (FBS), 10 mM HEPES, 1% nonessential amino acids, 1 mM sodium pyruvate and 10 lg/ml insulin. All other cell lines were obtained from American Type Culture Collection (Rockville, MD) and cultured according to conditions specified. Mammary organoid samples, kindly provided by Dr. Saraswati Sukumar (Johns Hopkins University School of Medicine, Baltimore, MD), were prepared from reduction mammoplasty specimens of women with no breast abnormalities. Breast tumor and bone metastasis tissues were obtained from the Surgical Pathology Division of the Johns Hopkins Hospital following the approval of the institutional review board (IRB) of the Johns Hopkins University School of Medicine. For all specimens, required written informed patient consents were obtained as approved by the IRB.

### Quantitative (q)RT-PCR

Total RNA was extracted using Trizol (Invitrogen) and cDNA was generated by reverse transcription. 25 μl reactions contained 1X SYBR Green Reaction Mix (Applied Biosystems), 1 μl cDNA, and 100 nm of each primer: Enpp1 (sense) 5′-GAAACGCCTCCTACCCTCTT-3′, (antisense) 5′-ATCCTGGCCAGAAAAATGTG-3′; GAPDH (sense) 5′-GTCAGTGGTGGACCTGACCT-3′, (antisense) 5′-TGCTGTAGCCAAATTCGTTG-3′. qRT-PCR parameters were: 1 cycle (95°C for 3 minutes) and 40 cycles (95°C for 30 seconds, 61.9°C for 30 seconds, and 72°C for 45 seconds). Amplification of GAPDH was used as an internal control. Relative expression between samples was calculated by the comparative C_T_ method.

### Western analysis

Total protein was extracted from cell lines using lysis buffer consisting of 15% glycerol, 5% SDS and 250 mM Tris-HCl, pH 6.7. Equal amounts of protein were resolved using 10% SDS- PAGE. Protein was transferred to ECL nitrocellulose membranes (Amersham) and probed with anti-Enpp1 (Everest Biotech) and β-actin (Sigma-Aldrich) antibody. Membranes were then incubated with horseradish peroxidase-conjugated antibody against rabbit IgG (Amersham) and binding was revealed by chemiluminescence (Amersham).

### Immunohistochemistry

Paraffin-embedded sections were deparaffinized in xylene and rehydrated through graded ethanol. Antigen retrieval was achieved by immersing sections in 0.01 mol/L sodium citrate (pH 6.0) and heating in a steamer for 20 min. Sections were cooled to room temperature (RT), and endogenous peroxidase activity was quenched by immersing in 0.3% hydrogen peroxide. Blocking was carried out by incubation in diluted normal rabbit serum (Vector Laboratories) as per the manufacturer's instructions. Sections were then incubated with goat polyclonal anti-Enpp1 (Everest Biotech) at a 1:750 dilution for 16 hours at 4°C. Diluted biotinylated anti-goat IgG (Vector Laboratories) was added to the sections and incubated for 30 min. at RT followed by Vectastain ABC reagent. Enpp1 proteins were visualized using 3, 3′-diaminobenzidine (DAB) as per the manufacturer's instructions (Vector Laboratories). Sections were subsequently washed in water and counterstained in hematoxylin (Richard-Allan Scientific). Images were acquired by light microscopy.

### Nucleotide Phosphodiesterase activity assay

Cells were plated in triplicate in a 96-well plate at 3000 cells/well and cultured in complete media for 72 hours. 1 μg/ml *p*-nitrophenylthymidine monophosphate was then added to each well as a substrate for phosphodiesterase and the reaction was allowed to proceed for 1 hour at 37°C. Formed *p*-nitrophenol was then quantified by measuring the absorbance at a wavelength of 415 nm in a microplate reader.

### In vivo assessment of bone metastasis and osteolysis

To determine the effect of Enpp1 on the establishment of bone metastasis, Enpp1 cDNA was cloned into the retroviral expression vector, pBabe-puro (Addgene plasmid 1764), and MDA-MB-231 cells were infected with pBabe-puro or pBabe-puro-Enpp1. Stable pools were selected in the presence of 1 µg/ml puromycin (Sigma-Aldrich) for one week.

In separate experiments, tumor cells were injected into the right tibia (2.5×10^4^ cells) and left cardiac ventricle (1×10^5^ cells) of 5-week-old female athymic nude mice (NCI-Frederick Cancer Research Facility). To monitor osteolysis, digital radiographic images were obtained once per week using a Faxitron MX-20 X-ray unit (Faxitron X-ray Corp.) and osteolytic area was measured using MetaMorph image analysis software (Meta Imag- ing Series version 6.1, Universal Imaging Corp.). The experiment was terminated at 4 weeks when there was marked tibial osteolysis with or without soft tissue extension of the tumor in any group. To assess tumor area, tibiae were harvested, fixed in formalin for 24 hours, and decalcified in 10% EDTA, pH 7.4 for 48 hours. Paraffin-embedded sections (5 μm) were generated laterally throughout the tibiae at 100 μm intervals. A minimum of five sections was stained with hematoxylin and eosin, and light microscopic images were acquired. The total area occupied by intraosseous and extraosseous tumor was then measured using MetaMorph image analysis software.
